# The AKT/mTOR Signaling Pathway Was Mediated through the LINC00514/miR-28-5p/TRIM44 Axis

**DOI:** 10.1155/2022/1889467

**Published:** 2022-09-23

**Authors:** Lin Wu, Xingmei Zhu, Runfeng Wang, Shukai Sun, Bo Ma, Zhiguo Zhang

**Affiliations:** ^1^Department of the Central Laboratory, The Second Affiliated Hospital of Xi'an Medical University, Xi'an 710038, China; ^2^Department of Pharmacology, Shaanxi University of Chinese Medicine, Xianyang 712046, China; ^3^Department of Neurosurgery, Tangdu Hospital, The Fourth Military Medical University, Xi'an 710039, China

## Abstract

**Objective:**

Increasing evidence has demonstrated the essential role of lncRNAs in tumorigenesis. LINC00514, a novel lncRNA, was reported to be a promoter of malignant behaviors in cancer, but in pituitary adenoma (PA), its biological functions remain unclear.

**Methods:**

Herein, we measured LINC00514 expression by RT-qPCR analysis which indicated a significant elevation of LINC00514 expression in human PA tissues. Moreover, the effect of LINC00514 silencing on PA cell proliferation and invasion was, respectively, examined by CCK-8 and transwell assays.

**Results:**

The results showed that LINC00514 deletion markedly inhibited PA cell proliferation and invasion. Besides, investigation on the molecular mechanisms showed that LINC00514 might function as an endogenous RNA (ceRNA) to sponge miR-28-5p and TRIM44 was mediated by LINC00514-derived miR-28-5p in PA cells. Furthermore, the AKT/mTOR signaling pathway was mediated through the LINC00514/miR-28-5p/TRIM44 axis.

**Conclusion:**

To sum up, we suggested LINC00514 as a novel therapeutic target for PA treatment.

## 1. Introduction

Pituitary adenoma (PA) is a common benign tumor in the sellar region of intracranial area, accounting for about 15% of central nervous system tumors, and its incidence is second only to meningiomas and gliomas in intracranial tumors. Its main manifestations are excessive pituitary hormone secretion, metabolic dysfunction (menopause, lactation, acromegaly, etc.), and tumor mass effect (headache, visual field changes, etc.) [1]. Due to the multidisciplinary, complex, and diverse clinical manifestations, the current mainstay is a multidisciplinary diagnosis and treatment method and an individualized and precise treatment plan for appropriate surgery, radiotherapy, or chemotherapy [2]. However, some pituitary adenomas invade the septum sellar, cavernous sinus, sphenoid sinus, blood vessels, nerves, etc. during the growth process, showing the biological characteristics of invasive growth [3]. After the tumor invades the surrounding bone, pituitary adenomas often form local infiltration of the sinus cavity or tight wrapping of blood vessels and nerves, resulting in difficult dissection of the tumor, high difficulty in total surgery, high postoperative neurological complications, and high residual tumor rate and the high recurrence rate, which bring challenges to the treatment of pituitary adenomas and are therefore called invasive pituitary adenomas. Although many aspects of the molecular mechanisms of tumor invasion have been studied, the reasons for the aggressive growth of pituitary adenomas remain unclear [4, 5]. The current study found that the main pathophysiology of invasive pituitary adenomas is a persistent state of cell proliferation and cell cycle disturbance [6]. Therefore, elucidating the molecular mechanism of invasive growth of invasive pituitary adenomas is particularly important for the prevention and treatment of invasive pituitary adenomas. Further exploration of its potential molecular markers and potential therapeutic targets will provide a research basis for early warning, early diagnosis, and early treatment of invasive pituitary adenomas.

In recent years, lncRNA (long noncoding RNA, long chain nonencoded RNA), as research hotspots, was found to be disordered in different types of cancer. The regulatory effect is related to the recurrence, metastasis, and progress of cancer. In previous studies, several lncRNAs have been confirmed to have correlation with PA, development and invasion in clinical specimens and cell function experiments. At the same time, with the increasingly complete technology of the transcription group sequencing technology (RNA-seq) and gene chip technology, more and more lncRNAs have been discovered, and a coexpression network involving a variety of lncRNA and mRNAs is established to further provide more convenience for in-depth research of pituitary tumors. Studies on the whole-genome sequencing technology show that a minority of the mammalian genome is in the protein-encoded regions while a majority of it belongs to noncoding RNAs (ncRNA) [7, 8]. lncRNAs, important members of the ncRNA family, are transcripts with limited or without protein-coding potential [9]. These transcribed RNA molecules have a variety of functions including RNA metabolism and chromatin remodeling [10–12]. Recently, increasing evidence has demonstrated the essential role of lncRNAs in tumorigenesis [13, 14]. For example, LINC00514, a novel lncRNA, was reported to be a promoter of malignant behaviors in many types of cancer [15–17]. Nevertheless, its biological role in PA remains unclear.

Herein, LINC00514 was found having an elevated expression in PA tissues and its deletion hindered PA progression. Moreover, LINC00514 interacted with miR-28-5p to regulate TRIM44 expression and promoted PA progression partially via the AKT/mTOR pathway.

## 2. Materials and Methods

The study and all amendments were approved by the appropriate ethics committee (NH-TY20200102). The study was done in accordance with the protocol, its amendments, and standards of Good Clinical Practice. All participants provided written informed consent before enrolment.

### 2.1. Tissue Specimens

42 pairs of PA tissues and matched normal tissues were collected from PA patients who were hospitalized at Tangdu Hospital, the Fourth Military Medical University (Xi'an, China) without any preoperative adjuvant therapies. All tissue samples were stored appropriately.

### 2.2. Cell Lines and Cell Culture

PA cell lines HP75 and GH3 were cultured in RPMI-1640 medium containing 10% FBS and incubated with 5% CO_2_ at 37°C in a humidified atmosphere.

### 2.3. RT-qPCR

TRIzol reagent was applied for RNA extraction, followed by RT-qPCR analysis with the following primers: LINC00514, 5′-GCTCAACATCTCACTTCTCCCAC-3′ (forward) and 5′-CCTTCAGTGTCTGGGAAAGAGAG-3′ (reverse); GAPDH, 5′-GGTATGACAACGAATTTGGC-3′ (forward) and 5′-GAGCACAGGGTACTTTATTG-3′ (reverse); miR-28-5p, 5′-GGTCCTTGCCCTCAAGGAGCTCACA-3′ (forward) and 5′-AGTGCCTGCCCTCCAGGAGCTCACA-3′ (reverse); U6, 5′-GCTTCGGCAGCACATATACTAAAT-3′ (forward) and 5′-CGCTTCACGAATTTGCGTGTCAT-3′ (reverse).

### 2.4. Western Blot

In RIPA buffer, cells were lysed with protease inhibitors. After quantification and electrophoration, protein was moved to PVDF membranes, followed by blocking, overnight incubation with related primary antibodies, and probing with appropriate secondary antibody. For detection of protein bands, enhanced chemiluminescence kits (Pierce, Rockford, IL, USA) were used.

### 2.5. Cell Transfection

From Thermo Fisher Scientific (Waltham, MA, USA), LINC00514-targeted shRNA (shLINC00514) and the relevant negative control shRNA (shNC) as well as miR-28-5p mimic/inhibitor and miR-NC were obtained. Lipofectamine 2000 was used for cell transfection and RT-qPCR analysis for efficiency confirmation.

### 2.6. Proliferation Assay

Cells (2 × 10^3^) were seeded into a 96-well plate and cultured for different time, followed by addition of CCK-8 reagent (Dojindo, Japan) and further incubation for 4 h. Microplate readers were used to measure the absorbance of each well.

### 2.7. Invasion Assay

For detection of cell invasion, transwell chambers were used. Followed by resuspending in serum-free culture medium, 1 × 10^5^ cells were placed in the upper chamber (with Matrigel coated) and 20% FBS in the lower chamber. 24 h later, the invaded cells were counted under a microscope after being fixed and stained.

### 2.8. Luciferase Reporter Assay

The miR-28-5p binding sites in LINC00514 and TRIM44 3′UTR were predicted using the TargetScan database. The reporter plasmids Wt-LINC00514, Mut-LINC00514, Wt-TRIM44 3′UTR, or Mut-TRIM44 3′UTR were constructed with pmirGLO vectors (Promega, Madison, WI, USA), followed by transfection with miR-28-5p mimics or miR-NC. 48 h later, luciferase activities were evaluated by corresponding assay kits (Promega).

### 2.9. Statistical Analysis

The normality of the sample was determined with the Shapiro–Wilk test. Descriptive statistical data were evaluated with the exploratory analyses of the Tukey test. Quantitative mean data (PES/WES, ISQ, and B.L.) were assessed with the nonparametric Wilcoxon-Mann–Whitney *U* test to analyze the inferential statistical.

Each experiment was independently repeated three times, with data shown as means ± standard deviation (SD). For statistical analysis, GraphPad Prism 5.0 software was used, and for difference comparison, Student's *t*-test or one-way ANOVA was used. *p* < 0.05 was considered statistically significant.

## 3. Results

### 3.1. LINC00514 Expression Is Elevated in PA Tissues

To make clear the specific role of LINC00514 in PA, we examined its expression by RT-qPCR in 42 pairs of PA and matched normal tissues. The analysis suggested a much higher expression of LINC00514 in PA tissues than the normal tissues (Figure 1).

### 3.2. Silencing of LINC00514 Hinders PA Cell Proliferation and Invasion

Before further exploration on the functions of LINC00514 in PA, LINC00514 expression was silenced in HP75 and GH3 cells by shRNA transfection, and transfection efficiency was confirmed by RT-qPCR (Figures 2(a) and 2(b)). Thereafter, the impact of LINC00514 deletion on cell proliferation was evaluated by CCK-8 assays which suggested that the proliferation rate of HP75 and GH3 cells was markedly reduced by shLINC00514 transfection (Figures 2(c) and 2(d)). Meanwhile, the results from transwell assays showed that LINC00514 deletion impaired HP75 and GH3 cell invasion (Figures 2(e) and 2(f)).

### 3.3. LINC00514 Is Targeted and Negatively Mediated by miR-28-5p

It is well known that cytoplasmic lncRNAs could function as ceRNAs to be a sponge of miRNAs and thereby mediate the expression of miRNA targets at a posttranscriptional level [18, 19]. A previous study has identified that LINC00514 was mainly located in the cytoplasm [20]. Thus, we verified whether LINC00514 served as a sponge of miRNA during PA development. The bioinformatics analysis was applied to predict the target miRNAs of LINC00514, and among all candidates, miR-28-5p ranked top with the predicted binding sites shown in Figure 3(a). By dual-luciferase reporter assays, their interaction was further verified, suggesting a reduction in luciferase activity in the LINC00514-Wt group (Figure 3(b)). Additionally, Pearson's correlation analysis showed a negative correlation between LINC00514 and miR-28-5p expression in PA tissues (Figure 3(c)). Moreover, RT-qPCR was applied to examine the changes in miR-28-5p expression after downregulation of LINC00514, and the observations proved a remarkable upregulation of miR-28-5p in HP75 and GH3 cells following LINC00514 knockdown (Figure 3(d)).

### 3.4. miR-28-5p Is Decreased in PA, and miR-28-5p Inhibitor Reverses the Impact of LINC00514 Deletion on PA

By RT-qPCR, miR-28-5p expression was detected in PA. The analysis indicated a much lower level of miR-28-5p expression in PA tissues than the normal tissues (Figure 4(a)). To validate the regulatory mechanism of LINC00514 in PA, a series of rescue assays were conducted. As shown by CCK-8 assays, deletion of LINC00514 suppressed HP75 and GH3 cell proliferation, which was rescued by treatment with miR-28-5p inhibitor (Figures 4(b) and 4(c)). We obtained similar results in the transwell assay (Figure 4(d)).

### 3.5. TRIM44 Is Manipulated by LINC00514-Derived miR-28-5p in PA Cells

A direct target of miR-28-5p, TRIM44, was predicted by the bioinformatics analysis, with corresponding binding sites shown in Figure 5(a). The interaction between them was verified by luciferase reporter assays indicating a significant reduction in luciferase activity of TRIM44-Wt by miR-28-5p mimics (Figure 5(b)). In addition, we found that LINC00514 downregulation significantly decreased TRIM44 expression in HP75 and GH3 cells while miR-28-5p downregulation increased TRIM44 expression in these cells (Figures 5(c) and 5(d)). All these observations proved that LINC00514 depended on miR-28-5p to regulate TRIM44 expression.

### 3.6. LINC00514 Inhibits the Activation of the AKT/mTOR Pathway

To elucidate the molecular mechanism beneath the LINC00514/miR-28-5p/TRIM44 axis, we detected in PA cells the activity of the AKT/mTOR pathway, a crucial player in cancer progression [21]. The results suggested that AKT/mTOR phosphorylation was markedly weakened by LINC00514 downregulation in HP75 and GH3 cells (Figures 6(a) and 6(b)). Furthermore, AKT/mTOR activation by the agonist IGF-1 attenuated the suppressive effect of LINC00514 deletion on HP75 and GH3 cell proliferation and invasion (Figures 6(c)–6(e)).

## 4. Discussion

PA is difficult to treat for its main origin from the anterior pituitary, a special growth location [22]. Pituitary adenoma is a common intracranial tumor occurring in the pituitary gland, with monoclonal origin. Its pathogenesis is complex, involving multiple aspects such as genetic mutation, epigenetics, oncogene/tumor suppressor gene, and cell cycle dysregulation. Pituitary tumors can be divided into noninvasive pituitary tumors, invasive pituitary tumors, and pituitary carcinomas according to their biological characteristics. PA has the biological characteristics of some malignant tumors, and it is easy to be misdiagnosed clinically, with high postoperative residual and recurrence rates and relatively poor prognosis. At present, in the research on the invasiveness of PA, related explorations at the level of genes, miRNAs, and proteins emerge in an endless stream, but its classification and pathogenesis are still unclear. The discovery of new markers to guide clinical diagnosis and even treatment has become an important research topic [23].. Thus, it is crucial to explore more effective approaches for PA treatment.

Increasing evidence has demonstrated that a majority of transcripts from the human genome are lncRNAs and their roles in cancer development have become a research hotspot in recent years [7, 8]. For instance, lncRNA BDNF-AS suppresses oesophageal cancer cell proliferation, invasion, and EMT [24]. lncRNA POU3F3 promotes proliferation and inhibits apoptosis of breast cancer [25]. Herein, we found the association of a newly identified lncRNA LINC00514 with PA progression. The study showed that LINC00514 expression was remarkably raised in PA and its knockdown hindered PA progression. Like us, Mi et al. reported that LINC00514 was distinctly upregulated in osteosarcoma and silencing of LINC00514 suppressed cell growth, colony formation, and metastasis [16]. Similarly, Han et al. suggested in pancreatic cancer a high expression of LINC00514 and its enhancing effect on cell proliferation and invasion [17]. All these observations suggested the oncogenic role of LINC00514 in cancer.

By acting as ceRNAs, lncRNAs exert their biological functions to affect cancer development [18, 19]. A previous study indicated the cytoplasmic location of LNC00514 in a subcellular fractionation assay [20], indicating the ability of LINC00514 to function in PA progression as a ceRNA. In our study, the target miRNAs of LINC00514 were predicted using the bioinformatics analysis and miR-28-5p ranked top among all candidates. The interaction between them was validated by luciferase reporter assays. Many studies have reported abnormal expression of miR-28-5p in cancers and its close association with lncRNAs during cancer development [26–29]. Herein, we found that miR-28-5p negatively regulated LINC00514, and miR-28-5p inhibitors reversed the influence of LINC00514 deletion on PA progression, indicating that the tumor-promoting impact of LINC00514 depended on miR-28-5p.

A potential target for miR-28-5p, TRIM44, was identified by the bioinformatics analysis, and the binding site at TRIM44 3′UTR was confirmed by luciferase reporter assays. Numerous studies have demonstrated the oncogenic role of TRIM44 in various cancers [30, 31]. We assumed that there was a “ceRNA network” among LINC00514, miR-28-5p, and TRIM44. Our study indicated that LINC00514 downregulation or miR-28-5p upregulation markedly reduced TRIM44 expression in PA cells. These observations demonstrated that LINC00514 depended on miR-28-5p to regulate TRIM44 expression. Previous studies have reported an interaction between TRIM44 and AKT/mTOR signaling in cancer progression [32, 33]. It is known that AKT/mTOR activation is frequent in cancer progression [21, 34, 35]. Herein, we demonstrated the involvement of AKT/mTOR in LINC00514-mediated PA progression. The results suggested that AKT/mTOR phosphorylation was remarkably attenuated by LINC00514 or TRIM44 knockdown but sharply enhanced by miR-28-5p overexpression in PA cells. Additionally, treatment with IGF-1 (AKT/mTOR agonist) reversed the inhibitory effect of LINC00514 silencing on PA progression.

lncRNAs are group of homogeneous ncRNAs > 200 nucleotides in size and ubiquitous transcription products mediated by RNA polymerase II. Although they maintain poor sequence conservation across species, lncRNAs do display conserved structures, suggesting their involvement in various biological functions. Many lncRNAs are considered as competing endogenous RNAs (ceRNAs) for miRNAs, which is one of the important mechanisms by which lncRNAs exert their biological functions. As evidenced, lncRNAs regulate gene expression at the epigenetic, transcriptional, and posttranscriptional levels through various mechanisms. The arrangement of miRNAs in the network and the number of their interconnections with other molecules greatly affect their function. The junctions of the network consist of miRNAs or mRNAs that play a major role in regulating the entire network. mRNAs are located in central locations with a higher density of target sites and have been evolutionarily chosen as the primary site of action for miRNA-mediated direct repression. LINC00514 is a newly discovered lncRNA, which is related to the regulation of biological behaviors such as proliferation, metastasis, invasion, and immune regulation. LINC00514 is located at chr16:2988256-3002016 and has three major long noncoding transcripts of 313 bp, 3385 bp, and 2216 bp. It is closely related to miRNA. For example, in TNBC, lncRNAARF6 overexpression leads to the loss of miR-145, which promotes cell invasion. The lncRNAROR, a reprogramming regulator, is a ceRNA of miR-145, resulting in competitive repression with ARF6 and loss of mature miR-145 expression. Therefore, we speculate that LINC00514 may function as a ceRNA by targeting specific miRNAs to mediate TNBC progression.

In conclusion, our study demonstrated an elevated expression of LINC00514 in PA tissues. Besides, LINC00514 deletion attenuated PA cell proliferation and invasion. Mechanically, the LINC00514/miR-28-5p/TRIM44 axis and the AKT/mTOR pathway were involved in the regulation of PA progression. Taken together, this study suggested LINC00514 for PA treatment as a novel therapeutic target.

## Figures and Tables

**Figure 1:** LINC00514 expression is elevated in PA tissues. LINC00514 expression in PA tissues was evaluated by RT-qPCR (*n* = 42). ^∗^*p* < 0.05.

**Figure 2:** Silencing of LINC00514 hinders PA cell proliferation and invasion. HP75 and GH3 cells were transfected with shLINC00514 or shNC, followed by detection of LINC00514 (a, b) expression, (c, d) cell proliferation, and (e, f) cell invasion. ^∗^*p* < 0.05.

**Figure 3:** LINC00514 is targeted and negatively mediated by miR-28-5p. (a) The predicted binding sites. (b) Confirmation of the interaction between LINC00514 and miR-28-5p. (c) Correlation between LINC00514 and miR-28-5p expression in PA tissues. (d) miR-28-5p expression was measured in HP75 and GH3 cells by the RT-qPCR analysis after LINC00514 silencing. ^∗^*p* < 0.05.

**Figure 4:** miR-28-5p is decreased in PA, and miR-28-5p inhibitor reverses the impact of LINC00514 deletion on PA. (a) Detection of miR-28-5p expression by RT-qPCR in PA and normal tissues (*n* = 42). (b–d) Evaluation of HP75 and GH3 cell proliferation and invasion. ^∗^*p* < 0.05.

**Figure 5:** TRIM44 is manipulated by LINC00514-derived miR-28-5p in PA cells. (a) The predicted binding sites. (b) Confirmation of the interaction between TRIM44 and miR-28-5p by luciferase reporter assays. (c, d) Assessment of TRIM44 expression in HP75 and GH3 cells by western blot after LINC00514 downregulation or miR-28-5p upregulation. ^∗^*p* < 0.05.

**Figure 6:** LINC00514 inhibits the activation of the AKT/mTOR pathway. (a, b) The protein expression of p-AKT, AKT, p-mTOR, and mTOR in HP75 and GH3 cells with different treatments was measured by western blot. (c–e) Evaluation of HP75 and GH3 cell proliferation and invasion, after treatment with or without IGF-1 (10 *μ*M). ^∗^*p* < 0.05.

## Data Availability

All data generated or analyzed during this study are included in this published article.
